# Attentional Mechanisms and Improved Residual Networks for Diabetic Retinopathy Severity Classification

**DOI:** 10.1155/2022/9585344

**Published:** 2022-03-24

**Authors:** Juan Cao, Jiaran Chen, Xinying Zhang, Qifeng Yan, Yitian Zhao

**Affiliations:** ^1^School of Information Science and Engineering, Chongqing Jiaotong University, Chongqing 400000, China; ^2^Ningbo Institute of Industrial Technology, Chinese Academy of Sciences, Ningbo 400000, China

## Abstract

Diabetic retinopathy is a main cause of blindness in diabetic patients; therefore, detection and treatment of diabetic retinopathy at an early stage has an important effect on delaying and avoiding vision loss. In this paper, we propose a feasible solution for diabetic retinopathy classification using ResNet as the backbone network. By modifying the structure of the residual blocks and improving the downsampling level, we can increase the feature information of the hidden layer feature maps. In addition, attention mechanism is utilized to enhance the feature extraction effect. The experimental results show that the proposed model can effectively detect and classify diabetic retinopathy and achieve better results than the original model.

## 1. Introduction

Diabetic retinopathy (DR) is a common chronic complication of the diabetic eye, which causes ischemia in the retinal capillaries, leading to vasodilatation and rupture, resulting in greater damage to the retina [1]. There are two stages of DR: nonproliferative and proliferative. In the nonproliferative stage, macular edema and local ischemia occur in the retina and lead to vision loss. With the prolongation of the disease, nonproliferative lesions tend to deteriorate into proliferative lesions, which cause microvascular proliferation, retinal hemorrhage, and blindness. Diabetic retinopathy is now prevalent in 2.6% of the world's population [2], a condition that occurs mostly due to the low priority given to the disease and the delay in treatment due to the lack of visibility of the DR lesion. Treatment at an early stage of the disease can greatly reduce the impact of DR on patients' health.

Currently, in the medical field, the process of DR diagnosis, which is quite expensive and time-consuming, is slow and complex, and the difference in the presence of retinal lesions in the three stages of early lesions in DR is not obvious, which often leads to misdiagnosis and other conditions by physicians. With the development of artificial intelligence, computer-aided medical systems [3] are gradually applied to detect medical diseases, which can be implemented by traditional machine learning algorithms or deep neural networks. Researchers can achieve end-to-end learning through convolutional neural networks, which helps them learn lesion features and diagnose new images afterward by simply using the lesion images and lesion categories as training data. Compared with machine learning, the algorithm can save the time of manual annotation of features and achieve higher diagnostic accuracy, which has great potential for research.

In this work, we propose a residual network with improved residual blocks incorporating an attention mechanism [4] based on the ResNet [5] model and integrated preprocessing of the images to accurately detect DR levels. The first part of this screening system is a preprocessing stage in which we perform weighted image fusion, grayscale, contrast enhancement, and resizing of the images to a uniform size. After that, we used the preprocessed images as training data to train the proposed model and used it for testing the model metrics in the test set. The experimental results show that the network model can achieve efficient automatic detection and classification of diabetic retinopathy, which is of great practical importance for the correct diagnosis of retinal diseases caused by diabetes.

## 2. Related Works

Owing to the increase in the hardware computing power and the development of artificial intelligence, machine learning and deep learning algorithms are widely used in the field of medical imaging, and a new way of diagnosis and treatment has been designed: the computer-aided medical system. For DR, automatic screening systems can provide ophthalmologists with a reliable diagnosis in order to carry out the next step of treatment, thus reducing human and material consumption in the treatment process.

### 2.1. Principle Component Analyst and Neuron Networks

In the early diagnosis of diabetic retinopathy, researchers used a comprehensive analysis of the physical indicators of patients to determine the type of lesion. Wu et al. [6] used principal component analysis (PCA) to downscale the patient's physical indicators to obtain a composite variable more suitable for lesion type prediction and used it to construct a logistic regression model. This method fully considers the physical indicators of patients, making the diagnosis results more practical, but it needs a lot of manpower for data analysis. In subsequent studies, some researchers have combined neural networks with principal component analysis for DR classification. Bhatkar et al. [7] output composite features through PCA and trained multilayer perceptrons and generalized a feedforward network to obtain the final DR lesion results; finally, 95% accuracy, 94.45% sensitivity, and 100% specificity are obtained. Compared with using PCA, it shows better detection accuracy, but manpower is still needed for data collection.

### 2.2. Machine Learning Algorithms

Machine learning algorithms are one of the commonly used methods in DR detection. This method does not need to analyze patient data but reuses manually designed components for lesion recognition. Singh et al. [8] proposed a computer-based automated hybrid technique for the detection of nonproliferative lesions and used a virtual support vector machine (SVM) for the classification of the lesion degree. 97.1% sensitivity and 98.3% specificity were obtained, but the small dataset used reduced the application value of the algorithm. Roychowdhury et al. [9] introduced a computer-aided screening system, which uses the MinIMas algorithm to extract the features of lesions and utilizes the AdaBoost algorithm to retain the features with more weight. Then, the features are used to train the Gaussian mixture model and the K-nearest neighbor classifier for DR lesion-type detection, and 100% sensitivity, 53.16% specificity, and 0.904 AUC are obtained. Compared with other advanced algorithms, it shows better performance but does not consider the detection of nonproliferative lesions.

### 2.3. Deep Learning Algorithms

The end-to-end deep learning algorithm can learn the features of the lesion image and its category and automatically screen the DR lesion category. Early researchers used simple models for detection tasks, which had high classification efficiency but poor classification performance. Pratta et al. [10] proposed a convolutional neural network model with a total of 12 layers and trained it with a large dataset of more than 80000 images. The model finally obtained 75% accuracy, 30% sensitivity, and 95% specificity. This method has strong generalization ability in lesion screening but does not achieve better detection results. Bodapati et al. [11] used the VGG16 [12] model for feature extraction, fused the feature maps of multiple specific layers and used them for final lesion detection, and finally obtained an accuracy rate of 84.31%.

Some researchers have improved the existing models for DR detection tasks. Shrivastava et al. [13] used the Inconcept V3 [14] network for feature extraction and used the extracted feature map to train the SVM classifier with a radial volume function and achieved 81.8% accuracy and 0.93 AUC. This method applies a network model with a complex structure for DR detection and improves the performance of the model. Fan et al. [15] proposed an adaptive weighted multiscale feature fusion neural network based on MobileNet V3 [16] and obtained 85.31% accuracy, 0.726 sensitivity, and 0.931 specificity on the APTOS 2019 dataset. This work introduced an adaptive weighted attention mechanism for feature fusion and improved the classification performance of the original model, but the small dataset used cannot guarantee the generalization ability of the model.

With the emergence of a variety of advanced neural networks, researchers can combine multiple models to obtain an integrated model. Compared with a single model, the integrated model has better experimental indicators but has higher requirements for experimental hardware. Jiang et al. [17] integrated ResNet 152 [5], Inception V3, and Inception-Resnet-V2 [18] for lesion detection of DR and obtained 88.21% classification accuracy, 85.57% sensitivity, and 90.85 specificity. Compared with a single model, the integrated model shows higher performance and robustness but increases the difficulty of training the model. Alyoubi et al. [2] proposed a CNN512 model and a YOLO V3 [19] model to determine the lesion grade by combining the DR detection results of the two models and obtained 89% accuracy on the DDR dataset, but the large volume of the CNN512 model limits the application scenarios.  Table 1 lists the datasets used in the above-mentioned works and their model evaluation indicators, including accuracy (ACC), sensitivity (SEN), and specificity (SP).

Compared with the above-mentioned methods, our proposed method has the following contributions: (1) The experimental results contain more comprehensive model evaluation metrics. (2) The use of open-source datasets provided by the Kaggle platform with a large data volume ensures the strong generalization ability of the model and its application value. (3) Deep learning algorithms are used for DR lesion screening without consuming a lot of human resources. (4) Compared with other advanced models, our method has better results in detecting the DR lesion stage. (5) By improving the original structure of the residual module and incorporating the attention mechanism, the proposed model has low requirements for experimental hardware and is easy to train the weight parameters of each layer.

## 3. Proposed Method

In this work, we aim to train several improved models using a data-enhanced and image-preprocessed fundus image dataset and select the best performing model. For the complex structure of retinal images and the inconspicuousness of lesions, it is often necessary to choose a neural network model with a more complex structure and a deeper network in order to improve the feature extraction effect. Therefore, we choose the ResNet network model as the backbone network and improve the feature utilization by modifying the structure of the residual blocks and introducing the attention mechanism [4]. The model structure is shown in Figure 1.

### 3.1. Backbone Network

ResNet is a deep network structure proposed by He et al. [5]. Compared with other network structures, ResNet uses a residual block to solve the problem of network degradation and gradient disappearance in the deep network; the residual block is shown in Figure 2, and a convolutional layer of 1 × 1 is used instead of 3 × 3 to perform the upscaling operation to reduce the computation so that the network depth is increased without degrading the performance. Let us consider *H*(*x*) as the feature of the next layer and *F*(*x*) as the output feature of the feature map calculated by the convolution layer, with *x* denoting the original feature map; then the relationship between F(x) and H(x) is as follows:

(1) $$\begin{array}{c} H\left(x\right)=F\left(x\right)+x. \end{array}$$

We adopt a shortcut connection in the residual block to feed the input feature *x* to the next layer. When the residue calculated by this layer is 0, we can still take the original feature *x* as the output so that the next layer can learn new features. Formally, in this paper, we consider a residual unit expressed as

(2) $$\begin{array}{c} \left\{\begin{array}{c} y_{l}=h\left(x_{l}\right)+F\left(x_{l},W_{l}\right),\\ x_{l+1}=f\left(y_{l}\right). \end{array}\right. \end{array}$$

Here, *x*_l_ and *x*_l+1_ are the input and output of the *l*th residual unit, respectively. The function *F*(*x*, *W*_1_) represents the learned features of the residual block, *h*(*x*_l_) = *x*_l_ is the constant mapping, and the function *f*(*y*_l_) is the activation function of the structure.

### 3.2. Improved Attention Mechanism

The convolutional block attention module (CBAM) [4] is formed by the channel attention module (CAM) [14] and the spatial attention module (Sam) [4] in series, and the feature map is processed by the CAM and SAM to obtain the features that retain important information in the channel and spatial dimensions. The weight matrix in the SAM is calculated from all the images in one batch; the dataset used in this paper utilizes data augmentation, and different sampling methods make the important features in each image be located differently. Hence, the weight matrix cannot integrate the information of all images well, resulting in the loss of features in the processed feature map and serious underfitting of the model in the experiment. The improved attention module is shown in Figure 3. The computation process of this module is as follows, where F is the input feature map and x_out_ is the output feature map of this module:

(3) $$\begin{array}{c} x_{\text{out}}=\text{CAM}\left(F\right)+\text{SAM}\left(F\right),\\ =M_{c}\left(F\right)\times F+M_{s}\left(\text{F}\right)\times F. \end{array}$$

In the CAM, the feature map *F* is input into the MLP network through a global pooling operation based on spatial dimension, the output feature map is fed into the MLP network, and finally, the add operation is performed and activated by the sigmoid function to obtain the channel attention feature; the output feature is obtained by multiplying the feature with the feature map F element by element. The CAM calculation process is as follows:

(4) $$\begin{array}{c} M_{c}\left(F\right)=\sigma \left(\text{MLP}\left(\text{AvgPool}\left(F\right)\right)\right)+\text{MLP}\left(\left(\text{MaxPool}\left(F\right)\right)\right). \end{array}$$

The feature map *F* is used as the input feature map of the SAM, and after the global pooling operation based on the channel, the output feature map is concatenated, and the spatial attention feature *M*_*s*_(*F*) is obtained by the convolution operation of the 7 × 7 matrix and the activation of the sigmoid function. The output feature is obtained by multiplying the feature map F element by element, and the calculation process is as follows:

(5) $$\begin{array}{c} M_{s}\left(F\right)=\sigma \left(f^{7\times 7}\left(\left[\text{AvgPool}\left(F\right);\;\mathrm{MaxPool}\left(F\right)\right]\right)\right), \end{array}$$

where *σ* is the sigmoid activation function and *M*_*s*_(*F*) is the weight matrix of the spatial dimension of the feature map *F*.

### 3.3. Residual Block

Before inputting the images into the model, the pixel values need to be normalized to float variables that are easier to handle by the GPU. We find that the values of the elements in the feature matrix obtained from the deeper layers of the network become very small after the normalized image is input into the model, which results in a large amount of missing feature information in the feature map processed by the attention mechanism, and thus, the input feature map needs to be enriched with information. In the following, we propose a solution to this problem from three aspects.

#### 3.3.1. Activation Function

The residual block structure in ResNet uses the ReLU activation function. When the input is negative, the output of the ReLU function is 0, and its first order derivative is also 0, which causes the death of neurons in this function, resulting in partial loss of feature information in the feature map. Therefore, all activation functions in the network are replaced with leaky ReLU activation functions, which can use this part of the feature information and learn it so as to retrain the feature information useful for classification. The expression of leaky ReLU is as follows:

(6) $$\begin{array}{c} f\left(x\right)=\left\{\begin{array}{cc} x, & \mathrm{if}\;x>0,\\ \alpha \left(e^{x}-1\right), & \mathrm{if}\;x\leq 0. \end{array}\right. \end{array}$$

#### 3.3.2. Bottleneck Layer

The bottleneck layer in the ResNet structure uses three convolutional layers to implement the upscaling operation of the feature map. The number of output channels of the 3 × 3 convolutional kernel in the bottleneck structure are set as *n*, the number of output channels of the 1 × 1 convolutional kernel as *m*, and the number of output channels of the bottleneck structure as *c*. Chu et al. [20] demonstrated that when m/*n* is smaller, the residual block has more expression capability and less redundancy of the feature map, so we improve the dimensioning structure in the residual block. In the original structure, *c* = *m*; now, we reduce *m* so that *m* + *n* = *c*, and the output feature map of the bottleneck layer retains some of the feature information of the feature map before dimensioning; the improved attention mechanism is added to the residual block to enrich the feature information that can be extracted from the bottleneck layer. The structure of the improved residual block is shown in Figure 4.

## 4. Experiments

To confirm the performance enhancement effect of introducing the attention mechanism and improved residual blocks on multiclassification tasks, three architectures were constructed to detect diabetic retinopathy in five stages, which are the ResNet50 model, ResNet50 model with improved residual blocks, and ResNet50 model with the attention mechanism and improved residual blocks. We have thoroughly evaluated the proposed method and compared it to the existing state-of-the-art segmentation methods to demonstrate the superiority of our model in the classification of diabetic retinopathy.

### 4.1. Data Preparation

The dataset used in this experiment is from the diabetic retinopathy detection competition on the Kaggle platform, with retinal images provided by EyePACS. The dataset contains 35126 high-resolution retinal images, which are divided into five categories according to the stage of the lesion, with a small proportion of retinal images in the severe and proliferative lesion stage. Based on the existing dataset, the data volume was increased to 40000 through data augmentation, 35000 of which are taken as the training set and 5000 as the verification set and test set so as to test the generalization ability of the model to new data and adjust the hyperparameters in the model in real time so as to prevent overfitting. The data distribution is shown in Table 2.

Figure 5 presents a few example retinal images of different stages of diabetic retinopathy from the dataset, where Figure 5(a) shows a healthy retina, Figure 5(b) shows a mildly diseased retina, Figure 5(b) shows a moderately diseased retina, Figure 5(c) shows an image of a severely diseased retina, and Figure 5(d) shows an image of a proliferative-diseased retina.

### 4.2. Image Preprocessing

There are a few incomplete or all-black images in the dataset, and the original retinal image contains a large number of black edges without information, which need to be screened out in advance. First, the position of the optic disc is found by graying and edge detection, and the radius of the minimum surrounding circle is found to cut the optic disc. Second, most retinal images have uneven illumination. The image with balanced illumination is obtained by graying the original image, Gaussian filtering, and weighted image fusion [21]. Finally, because the sizes of pictures in the dataset are different, the dimensions of the images are all resized to 512 × 512 pixels. An example of the original image and the preprocessed image is shown in Figure 6.

### 4.3. Evaluation Metrics

The performance of the proposed method is evaluated based on accuracy (ACC), kappa score, *F*1-score, sensitivity (SEN), specificity (SP), and precision (PRE). The mean values of sensitivity, precision, and specificity of the model at multiple lesion stages are used as evaluation metrics. The number of true positives is set as TP, the number of false positives as FP, the number of false negatives as FN, and the number of true negatives as TN in the prediction results; then the evaluation indexes of each category are calculated as follows.

For multiclassification tasks, the most intuitive evaluation metric is the all-category accuracy rate, which is the ratio of the number of correctly classified samples to the total number of samples, and it is denoted as

(7) $$\begin{array}{c} \text{Accuracy}=\frac{\text{TP}+\text{TN}}{\text{TP}+\text{TN}+\text{FP}+\text{FN}}. \end{array}$$

Precision is the proportion of the number of samples predicted to be positive that are true positives, and it is denoted as

(8) $$\begin{array}{c} \text{Precision}=\frac{\text{TP}}{\text{TP}+\text{FP}}. \end{array}$$

Sensitivity is the proportion of true positive samples that are predicted to be positive, and a higher value indicates that fewer of the positive samples are missed; it is denoted as

(9) $$\begin{array}{c} \text{Sensitivity}=\frac{\text{TP}}{\text{TP}+\text{FN}}. \end{array}$$

Specificity indicates the proportion of true negative samples that are predicted to be negative, and a larger value indicates fewer false positives in negative samples; it is denoted as

(10) $$\begin{array}{c} \text{Specificity}=\frac{\text{TN}}{\text{TN}+\text{FP}}. \end{array}$$

Kappa score evaluates the consistency of the model's classification by comparing the model's predictions with the labeled true labels, and it is denoted as

(11) $$\begin{array}{c} \text{Kappa Score}=\frac{\text{Obsered Accuracy}-\text{Expected Accuracy}}{1-\text{Expected Accuracy}}. \end{array}$$

The F1 score is the summed average of sensitivity and precision, which is used for the comprehensive evaluation of the model, and it is denoted as

(12) $$\begin{array}{c} \text{F}1\text{ Score}=2\times \frac{\text{Sensitivity}\times \text{Precision}}{\text{Sensitivity}+\text{Precision}}. \end{array}$$

### 4.4. Configuration

The proposed network architecture is implemented using the Python language and the Pytorch framework. All experiments were conducted on an NVIDIA Tesla P100 GPU with 16 GB of memory. The initial learning rate of the neural network used in the proposed method is set to 3*∗*10^−4^. In our experiments, we used multiple sets of initial learning rates and found that the convergence rate of the model decreases fastest when the learning rate approaches 1*∗*10^−4^. In our experiments, we found that the convergence of the model was slower after every 80 epochs, so we set the learning rate decay period to 80 epochs and the decay rate to 0.5. The proposed model was trained close to 270 epochs, and the loss function was nearly smooth, so we set each model to train 300 epochs to evaluate the test results of the model. To prevent the model from overfitting in the later stage of training, *L*2 regularization is added to the loss function of the model, and the regularization parameter is set to 1*∗*10^−3^ to prevent difficulties in training the model. In this experiment, DR lesion detection is a multiclassification task, so the cross-entropy function is used as the loss function, and the Softmax classifier is chosen as the classifier. The expression of the cross-entropy function is shown as follows:

(13) $$\begin{array}{c} L=\frac{1}{N}\sum_{i}L_{i}=-\frac{1}{N}\sum_{i}\sum_{c=1}^{M}y_{ic}\text{log}\left(p_{ic}\right). \end{array}$$

Here, *M* is the number of categories, *y*_*ic*_ is the conformity function, which takes 1 when the true category of sample *i* is *c*; otherwise, it takes 0, and *p*_*ic*_ denotes the predicted probability that the observed sample *i* belongs to category *c*.

## 5. Experimental Results

We have thoroughly evaluated our three constructed convolution neural networks and compared them to existing state-of-the-art classification methods in references [2, 11, 13, 15]. The evaluation results are shown in Table 3.

We used the three constructed convolution neural networks for training and testing the preprocessed dataset. Table 3 shows the experimental results of our three constructed network frameworks and other SOTA algorithms. The results show that the ResNet model with the improved residual block shows a small improvement over the original model in each metric because the improved residual block can provide richer image features to the Softmax classifier to improve the detection of lesion stages. Our proposed model performs better than ResNet and ResNet with the improved residual block in the task of DR lesion classification, and we believe that the improved attention mechanism makes full use of the feature maps containing more information, which enables the classifier to make better judgments. The special structure of the residual block makes the model structure deeper, and the feature maps in the deeper layers of the network have a higher field of perception so that the model can learn the feature information that cannot be perceived by the shallow network better.

Figure 7 presents the confusion matrix of our model and ResNet for the lesion classification task, with the true labels on the vertical axis and the model predictions on the horizontal axis. We can see that some of the images in categories 1, 2, and 3 are incorrectly classified into other categories; this is because the difference between the undiseased retina and the retina at the beginning of the lesion is small, but most of each category is classified as the true category. Both proliferate DR and severe DR were correctly classified, indicating that the problem of unbalanced data volume of each category in the original data is solved through data augmentation, and the model has learned the lesion characteristics of these two categories well.

The accuracy curves of the proposed model and ResNet are shown in Figure 8. It shows that the two models converge gradually after more than 200 epochs of training; in addition, the accuracy rates stabilize in the validation set, but the accuracy curves of the proposed model still have small fluctuations, which we believe is due to the instability of each value in the weight matrix output by the attention mechanism. After training, our proposed model can achieve a maximum classification accuracy of 91.3%, which is 2.9% better than that of the original model.

Table 4 shows the assessment metrics of our proposed model applied to each category in the diabetic retinopathy class classification task. Our proposed model achieves 0.893 on the kappa score, indicating that the predicted classification results of the model are in good agreement with the actual results. In addition, the *F*1 score reached 0.912, indicating that the model has high confidence in the identification results of lesions at all stages.

## 6. Discussion

In this work, we propose a ResNet network based on improved residual blocks and the attention mechanism for DR screening, which achieves satisfactory performance on the Kaggle dataset and provides an idea of how to apply the attention mechanism to medical images for feature extraction and improvement of datasets containing data with different distributions. The experimental results show that our proposed model achieves better classification results on the preprocessed dataset and a large number of images from the Kaggle dataset are utilized for model training to ensure the generalization and robustness of the model. Compared with some other SOTA algorithms, our proposed model shows better performance.

In addition, we found that using the attention mechanism directly to replace the original residuals or adding them outside the residual blocks caused the model to underperform the original model. We believe that the global pooling operation used by the SAM in calculating the weight matrix combines the feature importance of all images in one batch while the images are rotated after data augmentation so that the feature information is distributed differently; in addition, the output feature maps of the attention mechanism often contain less information. Therefore, the CAM is more suitable for this kind of task, and the model can perform better by connecting the channel attention mechanism and the spatial attention mechanism in parallel to achieve the complementary information of the two feature maps.

Table 4 shows that the improved model clearly performs better in the severe and proliferative DR categories, which is caused by the highest percentage of data-enhanced images in these two categories. For instance, the number of images in the severe stage in the source dataset only accounts for 2.4% of the total dataset, and the number of images in the proliferative stage is 1.8% of the total dataset, which greatly limits the ability of the model to diagnose lesions in these two stages and is more prone to overfitting. In order to solve the problem of data imbalance in the original dataset, data augmentation is an essential method, but the contrast in noise points increases with the enhancement of image features, which is detrimental to the classification of lesion stages. With the development of hardware computing power, a new trend in the field of diabetic retinopathy stage discrimination has emerged: multi-model integrated discrimination of the lesion level. For example, Liang et al. [22] trained AlexNet [23], ResNet50, and VGG16 to discriminate the lesion stage, and the final result was 79% accuracy by combining the three discriminations.

In the course of our work, we think the proposed method still has some shortcomings: (1) The dataset used in the proposed method is based on preprocessing operations such as Gaussian filter transform and weighted image fusion, and there is a small decrease in the detection accuracy when the unpreprocessed fundus images are detected. (2) The ResNet 50 network structure contains a large number of residual modules, which provide the input feature maps for the deeper layers by short-circuiting the connections but at the same time occupy some additional memory, thus imposing certain requirements on the equipment used, and further research on the optimization of the model is still needed in the future. (3) The image data to be detected should have the same data distribution as the dataset used in the experiment when the proposed model can achieve the best screening effect.

In the future, we can use a network suitable for discriminating the three stages of no DR, mild DR, and moderate DR to perform a comprehensive screening with the proposed model and improve the convolutional layers in the proposed model such as using asymmetric convolution instead of normal convolutional kernel to deepen the network while improving the efficiency of the model and increase the size of the input image to make the image details clearer. Further training and tuning of the system on a more balanced dataset should further improve the performance of the model.

## 7. Conclusion

Using an effective neural network-based screening system and scanner for regular scanning and diagnosis is beneficial for the mitigation and treatment of ocular diseases in diabetic patients. In this study, we proposed an effective and stable lesion severity classification model for the diabetic retinopathy classification task. By modifying the upper sampling level and residual structure of ResNet, we can get richer feature maps and use them for feature extraction of the attention mechanism. Thus, the feature map containing more important information can be used for the classification task of the classifier. An accuracy of 0.913, F1 score of 0.912, and kappa score of 0.893 were achieved, which are 2-3% higher than those of the original model and have demonstrated some potential for application in actual lesion diagnosis. Recent research in this area has shown a trend of combining image segmentation algorithms with image classification algorithms to improve model performance. In the future, this study will be expanded to other deep learning models combing image segmentation algorithms, and more datasets will be employed to achieve data balance and improve the generalization ability of the models.

## Figures and Tables

**Figure 1:** Architecture of ResNet.

**Figure 2:** Improved residual block structure.

**Figure 3:** Improved convolution block attention module.

**Figure 4:** Improved residual block structure.

**Figure 5:** Different categories of DR severity images. (a) No DR. (b) Mild DR. (c) Moderate DR. (d) Severe DR. (e) Proliferate DR.

**Figure 6:** Retinal images. (a) Original retinal image. (b) Processed retinal image.

**Figure 7:** Confusion matrixes for the severity prediction task. (a) ResNet50. (b) Proposed.

**Figure 8:** Accuracy curve of models. (a) ResNet 50. (b) Proposed.

**Table 1:** Summary of related works.

Method	Number of classes	Dataset	Performance measure			Limitation
			ACC	SEN	SP	
Wu et al. [6]	3	Private dataset	–	–	–	High manpower requirements
Bhatkar et al. [7]	2	Private dataset	–	1.0	0.5316	
Singh et al. [8]	4	DRIVE and STARE	–	0.971	0.983	Small dataset used
Roychowdhury et al. [9]	2	DIARETDB1&Messidor	94.23%	0.909	0.957	Proliferative lesions were not considered
Pratta et al. [10]	5	Kaggle	85.32%	0.726	0.931	Low screening accuracy
Bodapati et al. [11]	5	APTOS 2019	84.31%	–	–	Weak generalization capability
Shrivastava et al. [13]	5	Kaggle	81.8%	0.802	0.932	No complete model evaluation
Fan et al. [15]	5	APTOS 2019	85.32%	0.726	0.931	Small dataset used
Jiang et al. [17]	5	Private dataset	88.21%	0.855	0.908	Difficulty of training model
Alyoubi et al. [2]	5	DDR and APTOS 2019	89.0%	0.89	0.973	Huge model structure

**Table 2:** Retinal image data distribution.

Dataset	DR severity				
	No DR	Mild	Moderate	Severe	Proliferate DR
Training set	7000	7000	7000	7000	7000
Test set	1000	1000	1000	1000	1000

**Table 3:** Comparison between the proposed models and the state-of-the-art model.

Model	Performance measure					
	ACC (%)	F1 Score	Kappa score	SEN	SP	PRE
Bodapati et al. [11]	84.31	–	–	–	–	–
Shrivastava et al. [18]	81.8	0.862	–	0.802	0.932	0.89
Fan et al. [15]	85.3	0.853	0.773	0.727	0.931	0.744
Alyoubi et al. [2]	89.0	0.849	–	0.89	0.973	0.812
ResNet50 [2]	88.4	0.882	0.859	0.884	0.971	0.881
ResNet50 (improved residual block)	88.9	0.889	0.865	0.889	0.972	0.89
Proposed	91.3	0.912	0.893	0.913	0.978	0.912

**Table 4:** The performance metrics of the DR stages.

Stage	Sensitivity	Specificity	Precision
No DR	0.801	0.959	0.832
Regent's canal	0.942	0.975	0.901
Moderate	0.823	0.964	0.853
Severe	0.996	0.999	0.985
Proliferate DR	1.0	0.997	0.987

## Data Availability

The datasets presented in this article are publicly available on the Kaggle platform and can be found in Diabetic Retinopathy Detection (https://www.kaggle.com/c/diabetic-retinopathy-detection).
